This article has been retracted.

# A Multiscenario Intelligent QoS Routing Algorithm for Vehicle Network

**DOI:** 10.1155/2022/3924013

**Published:** 2022-06-27

**Authors:** Shitong Ye, Shaojiang Liu, Feng Wang

**Affiliations:** ^1^Department of Data Science, Guangzhou Huashang College, Guangzhou 511300, China; ^2^Guangzhou Xinhua University, Dongguan 523133, China

## Abstract

Vehicular ad hoc network (VANET) is a key part of intelligent transportation system. VANET technology is very important for realizing vehicle-to-vehicle communication, remote control of unmanned vehicles, and early warning reception of road condition information ahead of time when external networks such as the Internet are limited. Aiming at the problems of uncertainty in vehicle mobility, uneven distribution of traffic density in road sections, and uncertainty in the road scene where the vehicle is located in VANET, a multiscenario intelligent QoS routing algorithm (MISR) for vehicle network is proposed. The algorithm analyzes a variety of vehicle network scenarios and discusses the routing methods used in scenarios with/without roadside auxiliary units and vehicle uniform acceleration limited/unrestricted, so that the vehicle network can ensure that the communication link is not interrupted as much as possible. At the same time, QoS performance criteria such as data transmission rate, bit error rate, and delay time are considered. For complex scenes with variable vehicle speeds, this paper introduces a deep reinforcement learning method to intelligently select routing nodes for vehicle networks.

## 1. Introduction

At present, the network architecture of the vehicle network is diversified. For example, the vehicle equipped with communication sensors can realize the vehicle self-organizing communication network, the vehicle can realize the local area communication network with the help of the roadside auxiliary unit, and the vehicle can realize the vehicle mobile Internet network through 3G/4G/5G technology. With the continuous increase of global per capita car ownership, the research and application of vehicle network has received more attention. In recent years, with the in-depth research of artificial intelligence technology and wireless communication technology, the development of vehicle network has been promoted to a certain extent [1, 2]. At present, international researchers and technical experts are continuously achieving innovative results in the study of driverless technology. In the future, intelligent transportation is expected to replace human-driven vehicles through high-speed computing and intelligent analysis of computers, and further ensure passenger safety [3, 4]. However, driverless technology is highly dependent on the Internet, so it is necessary to receive the early warning information of the road ahead in real time through the Internet, so that unmanned vehicles can conduct intelligent analysis in advance, make corresponding route change plans or adjust the driving speed in time, so as to avoid the road risk ahead. Once the 3G/4G/5G signals around the road are poor due to environmental constraints, the unmanned vehicle cannot receive the relevant early warning signals of the road ahead in time, which will affect the road early warning analysis of the unmanned vehicle [5, 6].

Vehicle-to-vehicle and vehicle-to-roadside auxiliary unit information communication forms are vehicle self-organizing network structures. At present, the vehicle self-organizing network is facing many challenges in research. For example, vehicles move fast, resulting in frequent network topology changes. The formed multihop connection has poor stability, and the quality of service is difficult to guarantee; vehicle nodes can only travel along the road, so the data packet transmission can only move forward in the direction of the road [7]. Since the vehicle self-organizing network adopts a multihop propagation method that relies on relay nodes, due to the frequent changes in the relative positions of nodes in the actual environment, when the amount of network data is large, individual nodes are often heavily loaded, resulting in longer delay time., and even packet loss [8, 9]. For this reason, this paper designs a multiscenario intelligent QoS routing algorithm for vehicle network by analyzing the network environment where the vehicle nodes are located, so that the vehicle network can construct the propagation route by comprehensively considering the communication interruption probability, node load, transmission delay, and other conditions, so as to efficiently complete the data transmission task.

## 2. Related Work

Some traditional wireless ad hoc network routing algorithms, such as AODV and GPSR, have been proved to be very effective in many network environments, but they cannot effectively adapt to the environment of VANETs. The main reason is that the network topology changes frequently due to vehicle mobility. If AODV, GPSR, and other routing methods are adopted, VANETs will have serious packet loss. As more and more scholars pay attention to the research field of vehicle self-organizing network, some new research results begin to come into being [10–13]. Li et al. propose a W-GPCR routing method for vehicular ad hoc networks, which first analyzes the relationship between vehicle node routes and other parameters, such as the Euclidean distance between node pairs, travel direction, and vehicle density. Secondly, a composite parameter weighting model is established, and a calculation method is designed for the existing routing problem. This method can adaptively select the weighted parameter ratio in different network scenarios to obtain the optimal next-hop relay node [14]. Rana et al. propose a link reliability-based multihop location-directed routing (MHDLR), which decides the next-hop node based on link reliability to create a strong persistent path from source to destination. In multihop VANET, the distance between vehicles directly affects the connectivity of vehicles. Therefore, in order to estimate the link reliability of vehicles, this method considers the distance and relative speed between vehicles and proposes a geometric-based positioning mechanism (g-blm) to estimate the vehicle spacing of vehicles. The performance of MHDLR estimates the routing indicators, namely path disappearance, message broadcasting time in the group, packet delivery rate, and throughput [15]. Mao et al. developed a target-driven and movement prediction (TDMP)-based routing protocol. The main idea of TDMP is to include the driver's destination target in the mobility prediction to assist the implementation of the routing protocol. Compared to existing georouting protocols that greedily forward packets to the next hop mainly based on their current location and partial road layout, TDMP considers intervehicle link state estimation to enhance packet transmission, as well as in fluctuating mobility and dynamic prediction of vehicle position in global road layout [16]. Zhi et al. proposed a vehicle path planning method for a dynamic road network based on travel time reliability, which classifies the running state of vehicles under the influence of downstream signal control according to distributed wave theory. The travel time of vehicles on the road segment is classified and predicted, and the travel time prediction value set is further transformed into the travel time reliability. For the vehicle route selection of a dynamic road network, the travel time reliability of the route determined by the product of the travel time reliability of the road segment is logarithmically transformed, and the Dijkstra algorithm is used to find the most reliable route as the target solution [17].

## 3. VANETs Scenario Analysis

When unmanned vehicles build VANETs on the road, a major challenge is how to construct efficient propagation routes according to the network scenarios they are in. For example, in some road scenarios, roadside auxiliary units are set on the roadside, and the source vehicle node can relay data through the roadside auxiliary unit and other vehicle nodes, so as to successfully transmit data to the destination node, without the network of roadside auxiliary units. The scene can only rely on other vehicle nodes for relaying. Due to the great impact of vehicle mobility on the routing efficiency of VANETs, in some road scenarios, the vehicle speed is not limited, the vehicle mobility changes greatly, and the communication interruption probability is large. However, in the speed-limited scenario, the change of vehicle speed is relatively controllable, and the interruption probability is relatively small. To this end, when studying the propagation routes of VANETs, we analyze different network scenarios where vehicles are located: scenarios with roadside auxiliary units, scenarios without roadside auxiliary units, scenarios with restricted vehicle speed uniform acceleration, scenarios with unrestricted vehicle speed uniform acceleration, and speed-variable scenarios, to select corresponding propagation routes for different vehicle scenarios to transmit data.

### 3.1. Analysis of Network Scenarios with Roadside Auxiliary Units

Figure 1 shows a VANETs scenario with a roadside auxiliary unit (RSU). In this scenario, the vehicle node can connect with the RSU within its wireless sensing range. When there are no other vehicle nodes around the vehicle node that can relay data, Roadside assistance units can be selected to relay data. When there are other vehicle nodes around the vehicle node that can relay data, whether the auxiliary unit or the vehicle node is selected to relay data is selected according to the routing criteria. Since the energy situation of the roadside auxiliary unit is sufficient, this network scenario does not consider For energy loss and energy load issues, the transmission rate and transmission error rate are comprehensively considered. At the same time, since the vehicle node can also select RSU to relay data when there are no other vehicle nodes available to relay data, the speed of the vehicle is not considered in this scenario. For example, in Figure 1, it is assumed that the vehicle (node 1) needs to transmit N data packets with a data size of N to the vehicle (node 3). Node 1 can select the RSU node for relaying, or node 2 for relaying data. In the figure, Rs is uniformly expressed as the communication radius of vehicle nodes, and Ru is uniformly expressed as the communication radius of RSU.

In this network scenario, the rate of data transmission is defined as

(1) $$\begin{array}{c} {\text{rate}}_{i}=\frac{W}{N_{i}}\log_{2}\left(1+\frac{P_{i}\delta_{i}}{N_{0}}\right). \end{array}$$

Among them, the subscript *i* represents the vehicle node or roadside auxiliary unit, *W* is the bandwidth of the wireless channel, *N*_*i*_ is the size of the transmitted data packet, *P*_*i*_ is the transmission power of the transmitted data, *δ*_*i*_ is the channel gain in the wireless channel, and *N*_0_ is the Variance of complex Gaussian channel white noise.

The transmission error rate from node *i* to node *j* is defined as

(2) $$\begin{array}{c} ER_{ij}=\left(\frac{1}{2}-\frac{1}{\sqrt{\pi }}e^{-\eta d_{ij}\varsigma }\right)\sqrt{10\;\log_{10}\left(\frac{P_{r,j}}{P_{t,j}-P_{r,j}}\right)}. \end{array}$$

Here, *ς* represents the path fading factor, *d*_*ij*_ represents the transmission distance, *η* represents the ground reflection coefficient, *P*_*r*,*j*_ represents the received power of the node *j*, and *P*_*t*,*j*_ represents all the energy received by the node *j*, including noise.

In the scenario of VANETs with roadside auxiliary units, the QoS routing criterion for node *i* to select the next-hop relay node *j* is expressed as

(3) $$\begin{array}{c} Q_{j}=\frac{\sqrt{P_{j}}}{2}\frac{{\text{rate}}_{i}}{\text{delay}\left(i,j\right)ER_{ij}}. \end{array}$$

Where in node *i* and node *j* may be vehicle nodes or roadside auxiliary units, *P*_*j*_ represents the transmit power of node *j*, and delay(*i*, *j*) represents the total waiting time for node *j* to receive data after data arrives at node *j*. According to the standard of *Q*_*j*_, node *i* comprehensively considers the transmission rate and transmission error of the next hop, as well as the transmit power of the next-hop node.

### 3.2. Analysis of Network Scenarios without Roadside Auxiliary Units

Figure 2 shows the VANETs scenario without RSU. Since the vehicle nodes do not have the cooperation of auxiliary units, they need to relay data through other vehicle nodes, and the vehicle speed needs to be adjusted so that the communication link of the vehicle nodes will not be interrupted before the data transmission is completed as far as possible. Therefore, in the scenario of VANETs without RSU, the communication interruption probability is first considered, and then the vehicle node load, transmission rate, and transmission error rate are considered.

In the absence of RSU assistance, intervehicle nodes need to be connected to each other to establish a communication link, so vehicle speed needs to be considered. In some road scenarios, vehicle speed acceleration is limited, such as on urban roads and highways, which are restricted by traffic rules. On some roads, vehicle acceleration is unrestricted, such as driving vehicles in the open field in the wild, vehicle communication networks during certain military exercises or wartime conditions. Therefore, in the network scenario without the roadside auxiliary unit, it is also necessary to consider the network situation when the uniform acceleration of the vehicle speed is limited and the uniform acceleration of the vehicle speed is not limited.

#### 3.2.1. Scenarios with Limited Speed and Uniform Acceleration

In order to successfully transmit the data packet of size *N*_*i*_ to the target vehicle node, the vehicle node *i* needs to select a candidate vehicle node that can meet the communication duration within the communication radius of the vehicle node *i*, and then select a vehicle node from the candidate vehicle nodes according to the QoS standard. The vehicle node acts as the best next-hop node. In the scenario where the vehicle speed is limited by constant acceleration, it is assumed that the speed of the vehicle cannot exceed *v*_Ε_, the time required to complete the transmission of a data packet of size *N*_*i*_ is *t*_*i*_, the coordinate of node *i* is (*x*_*i*_, *y*_*i*_), the initial speed is *v*_*i*_, the acceleration is *a*_*i*_, and the coordinate of *j* is (*x*_*j*_, *y*_*j*_), the initial velocity is *v*_*j*_, and the acceleration is *a*_*j*_. As shown in Figure 3, the communication duration between the vehicle node and its adjacent node *i* within the communication radius *Rs* is defined as

(4) $$\begin{array}{c} T_{ij}=\frac{Rs}{R_{ij}}\;t_{i},\\ R_{ij}=\left(\left(v_{i}t_{i1}+\frac{1}{2}a_{i}t_{i1}^{2}+v_{E}t_{i2}^{2}\right)-\left(v_{j}t_{j1}+\frac{1}{2}a_{j}t_{j1}^{2}+v_{E}t_{j2}^{2}\right)\right)\cos\;\theta_{1}+\sqrt{{\left(x_{i}-x_{j}\right)}^{2}+{\left(y_{i}-y_{j}\right)}^{2}},\\ t_{i1}=\frac{v_{E}-v_{i}}{a_{i}},t_{i2}=t_{i}-t_{i1},\\ t_{j1}=\frac{v_{E}-v_{j}}{a_{j}},t_{j2}=t_{i}-t_{j1}. \end{array}$$

Within the communication radius *Rs*, the vehicle node *i* will select the node *j* of *T*_*ij*_ ≥ *t*_*i*_ as the candidate next-hop node to form a candidate node set *A*, and then select the next-hop node from the set *A* according to the QoS criteria:

(5) $$\begin{array}{c} Q_{i}=\frac{\sqrt{P_{j}}}{2\;\log_{10}S_{j}+1}\;\frac{{\text{rate}}_{i}}{\text{delay}\left(i,j\right)ER_{ij}}. \end{array}$$

Among them, *S*_*j*_ represents the network load of the node *j*. Considering the network load of the node is because when a large number of data packets are transmitted on the road, the data packet queue of some vehicle nodes in key positions often becomes longer, causing buffer overflow, this will increase the probability of node packet loss. The network load *S*_*j*_ of node *j* can be expressed as

(6) $$\begin{array}{c} S_{j}=\min\left\{\frac{\sum_{k=1}^{K}b_{j,r}\left(k\right)}{\sum_{k=1}^{M}b_{j,t}\left(k\right)},1\right\}. \end{array}$$

*K* represents the number of times that node *j* receives data in the historical data of the network, *M* represents the number of times that node sends data, *b*_*j*,*r*_(*k*) represents the amount of data that node *j* receives data for the *k*-th time, and *b*_*j*,*t*_(*k*) represents the amount of data that node *j* sends data for the *k*-th time.

#### 3.2.2. Unrestricted Scene with Uniform Acceleration

In the scenario of unrestricted vehicle speed uniform acceleration, assuming that the vehicle acceleration has no upper limit, the communication duration between the vehicle node *i* and its neighbor node *j* within the communication radius *Rs* is defined as

(7) $$\begin{array}{c} T_{ij}=\frac{Rs}{R_{ij}}t_{i},\\ R_{ij}=\left(\left(v_{i}t_{i}+\frac{1}{2}a_{i}t_{i}^{2}\right)-\left(v_{j}t_{i}+\frac{1}{2}a_{j}t_{i}^{2}\right)\right)\cos\;\theta_{1}+\sqrt{{\left(x_{i}-x_{j}\right)}^{2}+{\left(y_{i}-y_{j}\right)}^{2}}. \end{array}$$

The same as the speed limit scenario, within the communication radius *Rs*, the vehicle node *i* will select the node *j* of *T*_*ij*_ ≥ *t*_*i*_ as the candidate next-hop node to form a candidate node set *A*, and then from the set *A*, according to formula (5), calculated *Q*_*i*_ to select the next-hop node.

## 4. Intelligent QoS Routing Algorithm under Variable Speed Conditions

In the vehicle network, for the scene without a roadside auxiliary unit, the front mainly considers the situation that the vehicle is moving forward under the condition of uniform acceleration, but for the situation where the vehicle speed is changeable, the previous method cannot be used for analysis, so the vehicle's speed sudden acceleration/deceleration conditions may result in link interruption. For this reason, based on the method of deep reinforcement learning, the network can learn through a large amount of data, so that the vehicle node can intelligently select the next-hop routing node according to the status of other vehicle nodes within the communication radius, and try to ensure that the link is not interrupted. Condition to improve network utility [18].

Assuming that there are *l* adjacent nodes within the communication radius of node *x*_*t*,*i*_, these nodes are represented by a set *X*={*x*_*t*+1,1_, *x*_*t*+1,2_,…, *x*_*t*+1,*l*_}, *t* represents the current time slot of node *x*_*i*_, *S*_*t*_ represents the current state of node *x*_*i*_, and *S*_*t*+1_ represents the next state. When the node *x*_*i*_ selects a node *x*_*t*+1,*j*_ from the set *X* as the next-hop node, it switches to the next state, and the value function obtained by the next state is

(8) $$\begin{array}{c} V\left(S_{t}\right)\leftarrow E_{\pi }\left[R_{t}+\gamma V\left(S_{t+1}\right)\right]. \end{array}$$

*R*_*t*_ is the payoff when reaching the next state, and *γ* is the discount factor. Where *R*_*t*_ after using *x*_*i*_ to select the next hop *x*_*t*,*j*_ is defined as

(9) $$\begin{array}{c} R_{t}=\left\{\begin{array}{cc} 0, & \text{when }d_{ij}>R_{s,}\\ VU_{ij}, & \text{when }d_{ij}\leq R_{s.} \end{array}\right.. \end{array}$$

That is, when the distance between node *x*_*i*_ and *x*_*t*,*j*_ exceeds *R*_*s*_, the benefit is 0, and when the distance between node *x*_*i*_ and *x*_*t*,*j*_ is always within the range of *R*_*s*_, the benefit of *VU*_*ij*_ is obtained, and *VU*_*ij*_ is related to the routing benefit, expressed as

(10) $$\begin{array}{c} VU_{ij}=w_{1}\text{delay}\left(i,j\right)+w_{2}\;ER_{ij}+w_{3}{\text{rate}}_{i}+w_{4}S_{j}, \end{array}$$

where *w*_1_, *w*_2_, *w*_3_, and *w*_4_ are normalized weight factors, and the weight value can be set according to the desired QoS standard.

In the vehicle network, the current node reaches the next state by selecting the action of the next-hop node. The Q-learning method is introduced. The Q value of the state action pair is stored in a table (q-table) and updated iteratively, so as to obtain the optimization process of the action value function:

(11) $$\begin{array}{c} Q\left(S_{t},a_{t}\right)\leftarrow Q\left(S_{t},a_{t}\right)+\alpha \left[R_{t}+\gamma \underset{a_{t+1}}{\max}Q\left(S_{t+1},a_{t+1}\right)-Q\left(S_{t},a_{t}\right)\right], \end{array}$$

where *α* is the learning rate and *γ* is the discount factor (attenuation coefficient).

A deep neural network is introduced for training, and a deep neural network is used to fit the *Q* function. Node *i* obtains the next state by selecting the next-hop node and obtains the corresponding routing benefits, and defines the loss function of the network in the training process as

(12) $$\begin{array}{c} L\left(\theta \right)=\frac{1}{2}{\left[R_{t}+\gamma \underset{a_{t+1}}{\max}Q\left(S_{t+1},a_{t+1},\theta \right)-Q\left(S_{t},a_{t},\theta \right)\right]}^{2}. \end{array}$$

Update the parameters according to the gradient *L*(*θ*)/*∂θ* until *Q*(*S*, *a*) converges.

## 5. Experimental Simulation Results

The experiment is carried out by simulation. The hardware configuration of the experimental platform is: Intel Core i7-11800H 2.30 GHz octa-core GeForce RTX 3080 GPU, 16G memory. The programming language uses Python, the deep learning framework uses PyTorch, and the target network environment is built on the OMNet++ discrete-time simulator to realize the interactive simulation of the two platforms. In the simulation experiment, the simulation environment includes a road with a length of 10 km and a width of 4 lanes, and there are two intersections at each end, so as to simulate a universal urban trunk expressway. The driving speed of the vehicles in the simulation environment is set to random generation mode, and the value range of the speed is 30∼80 km/h, and they all drive through the road in a free-flow state to generate the movement trajectory of the vehicle node, and import the trajectory file into OMNeT++ network simulation software for simulation experiments. The MAC sublayer protocol in the simulation environment is IEEE 802.11 DCF, the digital channel bandwidth is 2 Mbps, the vehicles are randomly distributed on the road in the initial state of the experiment, and the vehicle communication radius distance is set to 100 m, assuming that the nodes have sufficient computing power and the computing time is negligible, the set noise power is *P*_*c*_=1 × 10^−2^*W*, and the discount factor is *γ*=0.5.

In order to verify the effectiveness of the proposed method, it was tested with W-GPCR and MHDLR algorithms under the same experimental conditions and the results were compared and analyzed. In this experiment, the experimental comparison is mainly carried out in three aspects: the average number of interruptions of vehicle communication, the bit error rate of data transmission, and average delay time of data transmission. The experimental data results are the average of the results after 100 tests.

In order to test different scenarios of the vehicle network, the test is mainly carried out in two representative scenarios: (1) the experiment is carried out in the presence of roadside auxiliary units, and a roadside auxiliary unit is set every 1 km for a total of 10, and the communication coverage radius of each auxiliary unit is 200 m. (2) The experiment is carried out without the roadside auxiliary unit, the acceleration of the vehicle changes randomly every 10 s, the vehicle speed has no upper limit, and the lower limit is 0 km/h.

### 5.1. Scenarios with Roadside Assistance Units

The condition for the end of the simulation is that all vehicles leave the simulated road. In each simulation process, the number of vehicle nodes is changed, and the average number of vehicle communication interruptions under the condition of different vehicle nodes is obtained, as shown in Figure 4. It can be seen from the figure that as the number of vehicle nodes increases, the average number of vehicle communication interruptions of the algorithm gradually decreases. When the number of vehicle nodes reaches 40, the average number of vehicle communication interruptions is 0. When the source vehicle node is far from the roadside auxiliary unit and cannot be relayed through the roadside auxiliary unit, and the number of vehicle nodes is small, the source node cannot relay data through other nodes, and there will be a greater probability of communication interruption, so the number of interruptions increases. When the number of vehicle nodes increases to a certain extent, for example, the number of nodes in the figure increases to 30, the number of nodes that the source node can use to relay data in the network is large, and the probability of interruption is small. It can be seen from the figure that the method in this paper, when compared to the other two methods, had fewer interruptions occurred during the experiment.

Experiments are carried out on the average communication bit error rate of the vehicle network.

In this set of experiments, the source vehicle node and the destination vehicle node are randomly selected in the vehicle network with data of size 2 MB, and the bit error rate of transmitting the data from the source vehicle node to the destination vehicle node is counted. The results were taken as the average value, and the results in Figure 5 were obtained. Figure 5 shows the average communication bit error rate of the three algorithms in the vehicle network. From the results in Figure 5, it can be seen that with the increase of vehicle nodes, the communication bit error rate of the network gradually decreases, and when the number of vehicle nodes is small, the bit error rate is high. This is because when the number of vehicle nodes is small, the relay opportunities of the network are reduced, and the frequent communication link disconnection increases the transmission error of the network. From the comparison in the figure, compared with the W-GPCR method, the average bit error rate of this method is about 30% lower, and the average bit error rate is about 34% lower than that of the MHDLR method. Therefore, the method in this paper performs better than the other two methods in reducing the bit error rate.

In this set of experiments, the average communication delay of the vehicle network is tested. The system randomly selects the source node and the destination node, and the source node transmits 2 MB data to the destination node. The communication delay time is the time when the destination node successfully receives the data minus the time when the source node successfully sends the data, and it is stipulated that the source node will resend the data when the link is interrupted during the transmission process. A total of 100 experiments were carried out, and the communication delay time of 100 experiments was taken as the average delay time of network communication. It can be seen from the experimental results in Figure 6 that with the increase of the number of network nodes, the delay time will gradually decrease. This is because when the number of nodes is small, the link will be interrupted in the process of transmitting data from the source node to the destination node. The possibility of increasing the number of link interruptions will increase the total required time for the destination node to finally receive data. It can be seen from the comparison results in the figure that the MISR algorithm proposed in this paper can achieve better results in reducing the delay than the other two methods.

### 5.2. Scenarios without Roadside Auxiliary Units

Experimental tests are carried out in scenarios without roadside assistance units. This experiment is also to test the average number of vehicle communication interruptions under the condition of different numbers of vehicle nodes. It can be seen from the results in Figure 7 that, for the same number of nodes, in the scene without roadside auxiliary units, the average number of interruptions is higher than that in the scene with roadside auxiliary units. This is because, in the absence of roadside auxiliary units, the vehicle node can only be used for relay, and the vehicle node due to the instability of its movement process increases the probability of communication link interruption. In the case of roadside auxiliary units, the data relay process of vehicle nodes is more stable. It can be seen from the comparison results in the figure that the method in this paper has fewer communication interruptions than the other two methods in the absence of roadside auxiliary units and performs better in reducing the probability of communication interruptions.

Under the condition of no roadside auxiliary unit, 2 MB data are also used for the data transmission test, and the result after 100 experiments is taken as the average value, and the statistical result of bit error rate in Figure 8 is obtained. From the results in Figure 8, the bit error rate obtained in the experiment is higher than that in the scenario with the roadside auxiliary unit. This is because without the assistance of the RSU, the probability of interruption caused by relying on vehicle nodes to perform cooperative relaying is greater, thus increasing the probability of transmission errors. It can be seen from the results in the figure that the bit error rate of the method in this paper is reduced by about 60% compared with the W-GPCR method, and about 45% compared with the MHDLR method. Since the speed change of vehicle nodes is uncontrollable, the method in this paper introduces deep reinforcement learning to allow vehicle nodes to learn from a large number of vehicle scene data, intelligently select the next-hop node based on experience, reduce the probability of communication interruption and to obtain higher QoS benefits.

The test experiment of the average delay time of the network is carried out in the scenario without RSU cooperation, and the data packet with a size of 2 MB is also used as the data packet for transmission.  Figure 9 shows the average network delay without RSU. It can be seen from the figure that compared with the average network delay with RSU cooperation (Figure 6), the average network delay without RSU cooperation is larger. This is due to the lack of RSU cooperation which increases the probability of link outages. As the number of network nodes increases, the average network delay time decreases, and the increase in the number of nodes increases the probability of randomly distributed nodes finding a suitable relay node. It can be seen from the comparison in the figure that the MISR method proposed in this paper can still obtain a smaller average communication delay in the scenario without RSU cooperation.

## 6. Conclusion

Vehicle network routing has become a challenging research direction in the field of wireless communication networks due to the mobility, dispersion, and complex network environment of vehicle nodes. Aiming at the diversified vehicle network scenarios, this paper analyzes the possible network scenarios of vehicles and discusses the routing methods in the scenarios with roadside auxiliary units, no roadside auxiliary units, and limited and unrestricted uniform acceleration. For complex scenarios with variable vehicle speed, this paper adopts a deep reinforcement learning method to intelligently select the next-hop node, so that the vehicle network routing can better adapt to the complex situation of variable speed. It can be seen from the experimental comparison results that the MISR routing method proposed in this paper can play a better role in reducing the probability of communication interruption and reducing the bit error rate.

## Figures and Tables

**Figure 1:** Scenario model of VANETs with roadside auxiliary units.

**Figure 2:** Scenario model of VANETs without roadside auxiliary units

**Figure 3:** Connection diagram of nodes within the communication radius.

**Figure 4:** Average number of interruptions in vehicle-to-vehicle communication.

**Figure 5:** Network average bit error rate results.

**Figure 6:** Average network delay time.

**Figure 7:** Average number of interruptions in vehicle-to-vehicle communication without RSU.

**Figure 8:** Network average bit error rate results without RSU.

**Figure 9:** Average network delay time without RSU.

## Data Availability

The data used to support the results of this study needs to be obtained with the consent of the corresponding author.
